The article "Circ TYMP1 Inhibits Carcinogenesis and Cisplatin Resistance in Ovarian Cancer by Reducing Smad2/3 Phosphorylation via a MicroRNA-182A-3p/TGF1B Axis" was retracted in 2023. Reasons: signs of a paper mill; suspected computer-generated content; unreliable results or conclusions; concerns about the data.

# Circ TYMP1 Inhibits Carcinogenesis and Cisplatin Resistance in Ovarian Cancer by Reducing Smad2/3 Phosphorylation via a MicroRNA-182A-3p/TGF1B Axis

**DOI:** 10.1155/2022/1032557

**Published:** 2022-08-16

**Authors:** Yang Rao, Wenwen Zhang, Dan Li, Xiao Li, Yaomei Ma, Pengpeng Qu

**Affiliations:** ^1^Department of Gynecological Oncology, Tianjin Central Hospital of Gynecology and Obstetrics, Tianjin 300100, China; ^2^Research Institute of Obstetrics and Gynecology, Tianjin Central Hospital of Gynecology and Obstetrics, Tianjin 300100, China; ^3^Department of Gynecological Oncology, Tianjin Medical University Cancer Institute&Hospital, Tianjin 300100, China

## Abstract

TYMP1 is a cancer driver in several human malignancies. However, its significance in ovarian cancer (ovarian carcinoma) remains uncertain. This research aims to understand the TYMP1's role in ovarian carcinoma carcinogenesis and cisplatin (DDP) resistance and its molecular ovarian marchionesses. Circ TYMP1 overexpression in ovarian carcinoma samples led to an accelerated tumor stage. Bioinformatics identified miR-182A-3p as the TYMP1's target transcript. Circ TYMP1 functioned as a sponge for miR-182A-3p, lowering its inhibitory effect on TGF1B. Downregulating circ TYMP1 decreased A2780-Res cell proliferation, invasion, and death resistance. Malignant ovarian carcinoma cells recovered following miR-182A-3p downregulation. TGF1B overexpression boosted A2780-Res cell proliferation, aggression, and cisplatin resistance while reducing Smad2/3 phosphorylation. TYMP1 sequesters miR-182A-3p and promotes TGF1B in ovarian carcinoma, boosting carcinogenesis and cisplatin resistance. This might lead to novel ovarian carcinoma treatments.

## 1. Introduction

In 2018, 300,000 new cases of ovarian cancer were diagnosed, and 185,000 people lost their lives to the disease. The diagnosis of ovarian carcinoma is commonly delayed, resulting in a considerably increased risk of both metastasis and recurrence [1]. At five years, the advanced patient survival rate was thirty percent, whereas the rate at ten years was fifteen percent [2]. Patients with advanced ovarian cancer frequently get cisplatin (DDP) [3]. The therapy of ovarian carcinoma is made more difficult by recurrent tumors and established chemo-resistance [4]. Biomarkers or molecules that fight against ovarian carcinoma might result in the development of new treatments.

The transcription of RNAs originates from around 75% of the human genome [5]. Some researchers believe that competing endogenous RNA, often known as ceRNA, can bind to miRNA and reduce its effects [6]. This family of ceRNAs is widespread in animals and has been linked to disorders affecting humans [7]. Loop structures are produced when pre-mRNA's 5′ and 3′ ends are contently connected [8]. Ovarian carcinoma is characterized by more significant number of circular RNAs and interacts with other transcripts [9]. Through the ovarian carcinomas of back splicing, the oncogene known as Circ TYMP1 is produced in esophageal squamous cell carcinoma [10]. Circ TYMP1 has also been linked to an increased risk of developing cervical [11] and breast cancer [12]. The ovarian carcinoma role in the circ TYMP1 production is unknown. MiR-182A-3p has the ability to bind to TGF1B mRNA as well as circ TYMP1. MiR-182A-3p suppresses hepatovarian adenocarcinoma carcinoma [13]. The downregulation of miR-182A-3p in lung cancer cells lowers the cytotoxicity caused by cisplatin [14]. TGF1B's outlook in ovarian carcinoma is gloomy, according to [15]. It is yet unknown how TGF1B influences the development of ovarian carcinoma tumors or therapy resistance. A TYMP1/miR-182A-3p/TGF1B *axis* is involved in developing ovarian carcinoma tumors.

The article "Circ TYMP1 Inhibits Carcinogenesis and Cisplatin Resistance in Ovarian Cancer by Reducing Smad2/3 Phosphorylation via a MicroRNA-182A-3p/TGF1B Axis" was retracted in 2023. Reasons: signs of a paper mill; suspected computer-generated content; unreliable results or conclusions; concerns about the data.

## 2. Materials and Methods

### 2.1. Ethics Statement

Our hospital's Ethical Committee approved this study, which followed the Helsinki Declaration. Respondents signed permission forms.

### 2.2. Immunohistochemistry (IHC) Adenocarcinoma Staining

The dewaxed tissues were rehydrated in alcohol and sectioned at 4 m. The sections were then grown in 3% hydrogen peroxide (Sigma-Aldrich Chemical Company), boiled in 0.01 M citrate buffer and blovarian adenocarcinoma with goat serum working solution (PCN5000, Invitrogen, Thermo Fisher Scientific Inc., Waltham, MA, USA). The parts were then washed at room temperature. The slices were then treated with streptavidin-working solution (S-A/HRP, Innova Biosciences, Cambridge, UK, 2010-1000) at 25°C for 10 minutes. The slices were stained with diaminobenzidine for 8 minutes at 25 degree Celsius. Alternatively, hematoxylin counterstaining, dehydration, cleaning, sealing with neutral glue, and light microscopy are utilized (Nikon Instruments Inc., Tokyo, Japan). Image-Pro Plus was utilized to determine the quantity of IHC-positive cells in each sample (Nikon). The cytoplasm of positively labeled cells included brownish or tan granules.

### 2.3. MTT

Using the MTT technique, cell viability was evaluated. In 96-well plates, 103 cells were sorted, and six duplicate wells were set up for each group. After 12 hours, the cells were treated with increasing concentrations of cisplatin for another 48 hours. Each well was filled with 10 L of MTT (5 mg/mL, Sigma-Aldrich) and incubated at 37°C for 4 hours. The supernatant was then discarded, and 150 mL of dimethyl sulphoxide solution was added to each well (Sigma-Aldrich).

The article "Circ TYMP1 Inhibits Carcinogenesis and Cisplatin Resistance in Ovarian Cancer by Reducing Smad2/3 Phosphorylation via a MicroRNA-182A-3p/TGF1B Axis" was retracted in 2023. Reasons: signs of a paper mill; suspected computer-generated content; unreliable results or conclusions; concerns about the data.

### 2.4. TUNEL

Prepared slides were fixed in 4% PFA for 30 minutes before being penetrated with 0.1% Triton X-100 in 0.1% sodium citrate for 2 minutes. As instructed, the TUNEL kit (Rovarian carcinomahe Ltd., Basel, Switzerland) was utilized. Cells were labeled with 4′, 6-diamidino-2-phenylindole after 90 minutes of incubation at 37°C with 1 percent TdT enzyme (DAPI, Sigma-Aldrich). The TUNEL-positive cells were green under a fluorescent microscope, whereas the total number of cells appeared blue. Each group was assigned five fields of vision at random. (apoptotic cells/total cells) × 100%.

### 2.5. Transwell Assay

Before being detached, cells that had been stable after transfection were starved for twenty-four hours. Plates with 24 wells and transwell chambers Coatings of Matrigel (diluted at a ratio of 1 : 8, 356234, BD Biosciences, Franklin Lakes, New Jersey, USA) were applied to the apical chambers (diluted at 1 : 8, 356234, BD Biosciences, Franklin Lakes, NJ, USA). After being divided into their respective groups, the cells were washed and then resuspended in serum-free RPMI-1640. The basolateral chambers were filled with 600 liters of RPMI-1640 that included 20 percent fetal bovine serum, whereas the apical chambers were filled with 200 liters of cell suspension. The cells that invaded the bottom membrane were fixed in PFA at a concentration of 4% for 15 minutes and then stained with crystal violet at a concentration of 0.5% for 20 minutes.

### 2.6. Reporter Gene Assays

MiR-182A-3p mimic or mimic NC were cotransfected into 293T cells. After 48 hours, an assay method measuring dual-luciferase activity in cells was utilized (Promega).

### 2.7. FISH

Examining the subcellular lovarian carcinomaalization of circ TYMP1 in ovarian carcinoma cells with the use of an RNA FISH Probe Kit was one of the studies that was conducted (F11201, GenePharma Co., Ltd., Shanghai, China). It was particularly seeded in 24-well plates at a density of 6 104 cells per well. After doubling the cells in PBS, the samples were fixed in 1 mL of 4% PFA, treated with 2 g/mL proteinase K, glycine, and an acetylating agent and then incubated in 250 L of prehybridization solution at 42 degree Celsius for one hour. And that is it. After that, the cells were cultured for one more night at a temperature of 42 degrees Celsius in a hybridization solution containing probe at a concentration of 300 nanograms per milliliter. The nuclei of the cells were then stained with DAPI (1 : 800) for a period of 5 minutes. The cell slides were treated with a quenching chemical to prevent fluorescence from escaping.

### 2.8. RNA Pull-Down Assay

After the ovarian cancer cells were eliminated, the remaining cells were processed using centrifugation with 0.25 percent trypsin (Gibco). After placing the precipitates in RIP lysis buffer, the mixture was refrigerated and subjected to lysis for a period of five minutes. An RNA pull-down experiment was utilized in order to look into the possible binding interaction between circ TYMP1 and miR-182A-3p. This investigation was carried out in order to learn more about how these two molecules interact. During the previous night, biotin-labeled Bio-circ TYMP1-WT, Bio-circ TYMP1-MUT, and Bio-NC were used to treat cell lysates. These treatments were performed in the laboratory (RiboBio Co., Ltd., Guangdong, China). After that, the cell lysates were left out for forty-eight hours in an environment that included magnetic beads that had been coated with streptavidin (Invitrogen, Thermo Fisher Scientific). In order to investigate the amount of miR-182A-3p expression, real-time quantitative PCR was performed.

The article "Circ TYMP1 Inhibits Carcinogenesis and Cisplatin Resistance in Ovarian Cancer by Reducing Smad2/3 Phosphorylation via a MicroRNA-182A-3p/TGF1B Axis" was retracted in 2023. Reasons: signs of a paper mill; suspected computer-generated content; unreliable results or conclusions; concerns about the data.

### 2.9. RT-qPCR

RNA was extracted from cells and tissues using a miRNeasy Mini Kit (Qiagen GmbH, Hilden, Germany). GenePharma Co., Ltd. Created the circ TYMP1, miR-182A-3p, and TGF1B primers, according the Genebank database (Shanghai, China). A3500 reverse transcription device was utilized to convert RNA to cDNA (Promega). Next, real-time qPCR was performed using the 7500 Real-time PCR System (Applied Biosystems, Inc., Carlsbad, CA, USA).  Table 1 contains the sequences of the primers, with *β*-actin serving as the internal control using the 2-Ct method to analyze relative gene expression.

### 2.10. Western Blot Analysis

50 *µ*g of protein was then separated on 10% sodium dodecyl sulfate-polyacrylamide gel and transferred to polyvinylidene fluoride membranes (Millipore). After 2 h of blovarian carcinomaking in nonfat milk, membranes were incubated overnight at 4°C with primary antibodies against TGF1B (1 : 1,000, ab96099, Abcam), Smad2/3 (1 : 5,000, ab179461, Abcam), p-Smad2/3 (1 : 5,000, ab124956, Abcam), and *β*-actin (1 : 5,000, ab8227, Abcam) (1 : 20,000, ab6721, Abcam). Utilizing a Bio-Rad Image analysis equipment, enhanced chemiluminescence reagent was employed to evaluate protein blots (Bio-Rad). The relative protein level (relative to -actin) was assessed using ImageJ.

## 3. Results

### 3.1. Circ_TYMP1 Is Upregulated

Circ TYMP1 expression in ovarian carcinoma tissues was more significant than in neighboring tissues (Figure 1(a)). The TYMP1 expression was comparable in A2780, SKOV3, ES2 ovarian carcinoma, and IOSE80 cells (Figure 1(b)). A2780-Res cells also demonstrated a greater level of circ TYMP1 expression than A2780 cells (Figure 1(c)). Afterward, the clinical relevance of circ TYMP1 was evaluated. Patients were classified into two groups based on their TYMP1 expression levels: high (*n* = 14) and low (*n* = 11). An increased expression level of circ TYMP1 was related with an increase in lymph node metastases and advanced tumor stage.

The article "Circ TYMP1 Inhibits Carcinogenesis and Cisplatin Resistance in Ovarian Cancer by Reducing Smad2/3 Phosphorylation via a MicroRNA-182A-3p/TGF1B Axis" was retracted in 2023. Reasons: signs of a paper mill; suspected computer-generated content; unreliable results or conclusions; concerns about the data.

### 3.2. Silencing of Circ_TYMP1 Reduces Drug Resistance

A2780-Res cells' drug resistance to cisplatin increased, as did the half-maximum inhibitory concentration (IC50) (Figure 2(a)). A2780-Res cells were transfected with oe-circ TYMP1 or sh-circ TYMP1 to study circ TYMP1's function in drug resistance. By overexpressing circ TYMP1, the cisplatin resistance of A2780-Res cells enhanced, whereas it reduced by silencing circ TYMP1 (Figure 2(b)). MTT findings demonstrated that overexpression of circ TYMP1 in A2780-Res cells enhanced drug resistance, whereas downregulation of circ TYMP1 decreased drug resistance (Figure 2(c)).

With circ TYMP1 overexpression, the amount of A2780-Res cell colonies rose, but it reduced with circ TYMP1 downregulation (Figure 2(d)). The TUNEL test demonstrated that oe-circ TYMP1 decreased apoptosis in A2780-Res cells, whereas sh-circ TYMP1 enhanced it (Figure 2(e)). In addition, transwell test findings have demonstrated that overexpression of circ TYMP1 boosted invasion potential whereas downregulation of circ TYMP1 lowered invasion potential (Figure 2(f)).

### 3.3. 2circ_TYMP1 Sponges MiR-182A-3p in Ovarian Carcinoma Cells

StarBase and circBank predicted the miRNA targets of circ TYMP1 (Figure 3(a)). Previous studies revealed that miR-182A-3p was underexpressed in ovarian carcinoma and that its absence contributed to the development of tumors (PMID: 33099316; PMID: 29616112). Circ TYMP1 then targets miR-182A-3p in ovarian carcinoma to advance ovarian carcinoma. RT-qPCR demonstrated reduced miR-182A-3p expression in ovarian carcinoma tumor tissues relative to surrounding tissues (Figure 3(b)). Furthermore, the ovarian carcinoma cell lines exhibited reduced miR-182A-3p expression (Figure 3(c)). Additionally, the A2780-Res cells expressed less miR-182A-3p than the A2780 cells (Figure 3(d)).

The TYMP1 was predominantly sublovarian carcinomalized in the cytoplasm of A2780 cells, as shown by FISH (Figure 3(e)) and obtained the potential miR-182A-3p-circ TYMP1 binding sequence (Figure 3(f)). In 293 T cells, the miR-182A-3p mimic decreased the circ TYMP1-WT luciferase activity. The activity of luciferase was not affected in cells transfected with mimic NC or circ TYMP1-MUT (Figure 3(g)). The circ TYMP1 and miR-182A-3p fragments were considerably enhanced when coupled with anti-AGO2 compared to anti-IgG (Figure 3(h)). A2780 cells were additionally transfected for RNA pull-down using Bio-circ TYMP1-WT and Bio-circ TYMP1-MUT. Consequently, chemicals interacting with Bio-circ TYMP1-WT enriched miR-182A-3p, whereas Bio-circ TYMP1-MUT enriched just a short fragment of miR-182A-3p (Figure 3(i)). These results indicated that that TYMP1 can bind to miR-182A-3p.

The article "Circ TYMP1 Inhibits Carcinogenesis and Cisplatin Resistance in Ovarian Cancer by Reducing Smad2/3 Phosphorylation via a MicroRNA-182A-3p/TGF1B Axis" was retracted in 2023. Reasons: signs of a paper mill; suspected computer-generated content; unreliable results or conclusions; concerns about the data.

### 3.4. MiR-182A-3p Inhibition Restored A2780 Resistance

We then studied miR-182A-3p in A2780-Res cancer and treatment resistance cells. RT-qPCR showed miR-182A-3p reduction in A2780-Res cells transfected with miR-182A-3p inhibitor or sh-circ TYMP1 (Figure 4(a)). The drug resistance of A2780-Res cells was increased by miR-182A-3p silencing (Figure 4(b)).

MiR-182A-3p suppression increased A2780-Res colony formation (Figure 4(c)). Downregulation of miR-182A-3p lowered apoptosis in A2780-Res cells (Figure 4(d)). MiR-182A-3p reduction increased A2780-Res invasion in transwell testing (Figure 4(e)). A2780-Res cells become malignant after miR-182A-3p suppression (Figures 4(c)–4(e)). MiR-182A-3p inhibits sh-circ TYMP1 and increases A2780-Res cell resistance.

### 3.5. MiR-182A-3p Directly Binds to TGF1B

According to StarBase data, miR-182A-3p possesses TGF1B mRNA binding sites (Figure 5(a)). The luciferase experiment demonstrated that miR-182A-3p inhibits the activity of TGF1B-WT luciferase vector in 293T cells, but has no effect on TGF1B-MUT luciferase vector (Figure 5(b)).

Consequently, RT-qPCR and IHC labeling demonstrated that TGF1B mRNA and protein levels were higher in ovarian carcinoma tumor tissues than in surrounding tissues (Figures 5(c) and 5(d)). Similar patterns were seen in cells with increased TGF1B expression in ovarian carcinoma cell lines compared to IOSE80 cells (Figures 5(e) and 5(f)). A2780-Res cells also displayed increased TGF1B expression compared to A2780 cells (Figures 5(g) and 5(h)), showing that TGF1B may be responsible for ovarian carcinoma carcinogenesis and drug resistance through circ TYMP1/miR-182A-3p (Figures 5(i) and 5(j)). TGF1B mRNA and protein levels dropped during activation of miR-182A-3p but rose upon inhibition.

## 4. Discussion

Even though it is not the most common form of cancer affecting female reproductive organs, ovarian carcinoma has the highest percentage of fatalities [15]. Individuals diagnosed with advanced ovarian carcinoma had poor results, even after undergoing surgical debulking and receiving chemotherapeutic medications [16]. Ovarian cancer treatment challenges center on managing uncontrolled tumor growth, the spread of the disease to other parts of the body, and developing resistance to chemotherapy drugs. We discovered that circ TYMP1 increases the synthesis of TGF1B by sequestering miR-182A-3p. This reduces the amount of Smad2/3 phosphorylation, promoting carcinogenesis and cisplatin resistance in ovarian carcinoma cells. The researchers discovered that a significant amount of circ TYMP1 expression in the ovarian carcinoma cells and tissues. This particular circRNA can be found in high levels in various human cancers, including gynecologic tumors [11]. On the other hand, almost little is known about the role that circ TYMP1 plays in establishing ovarian carcinoma, particularly in relation to drug sensitivity [12]. According to our research findings, drug-resistant A2780-Res cells exhibit higher amounts of circ TYMP1 than drug-sensitive A2780 cells. As a result of being treated with cisplatin, A2780-Res cells saw a decline in their vitality, invasion, and resistance to death. These findings suggest that inhibiting circ TYMP1 has a tumor suppressive effect in ovarian carcinoma and that circ TYMP1 may be connected with cisplatin resistance in cancer cells. In addition, these findings suggest that circ TYMP1 may be involved in the development of ovarian carcinoma.

The article "Circ TYMP1 Inhibits Carcinogenesis and Cisplatin Resistance in Ovarian Cancer by Reducing Smad2/3 Phosphorylation via a MicroRNA-182A-3p/TGF1B Axis" was retracted in 2023. Reasons: signs of a paper mill; suspected computer-generated content; unreliable results or conclusions; concerns about the data.

It is well known that aberrant expression of miRNAs, which are now the noncoding RNAs that have received the most attention from researchers, and ceRNA sponges are related to cancer [12]. The luciferase unequivovarian carcinoma tests all established miR-182A-3p as TYMP1's target miRNA. MiR-182A-3p is a tumor suppressor that inhibits the growth and invasion of cancer cells [13]. It is particularly effective against hepatitis ovarian carcinoma cellular carcinoma and lung cancer. Significantly, downregulation of miR-182A-3p reduces the amount of apoptosis that ovarian carcinoma cars in ovarian carcinoma OVCAR3 and CAOV-3 cells while simultaneously promoting proliferation, migration, and invasion. We found that the expression patterns of miR-182A-3p in ovarian carcinoma tissues and cell lines were quite similar to one another. The drug resistance and malignant potential of A2780-Res cells, which this miRNA had previously reduced, were restored when the circ TYMP1 gene was silenced. Overexpression of miR-182A-3p increased the anticancer effects of cisplatin in lung cancer cells, as reported by Li et al. in a prior study [14]. There is a possibility that the downregulation of miR-182A-3p is responsible for the increased cisplatin resistance that is mediated by circ TYMP1.

The direct interaction between miR-182A-3p and TGF1B was demonstrated with the help of a luciferase experiment. TGF1B is abundant in the natural world and is thought to have a role in several different biological ovarian carcinomas [17], including the production of nucleic acids, carbohydrates, and proteins. TGF1B is present in high levels in tumors because the energy levels of rapidly dividing tumor cells are higher [17]. It was shown that ovarian carcinoma tissues had a considerable amount of TGF1B expression, and increasing the amount of TGF1B expression in ovarian carcinoma cells increased their viability [15]. It has been discovered that TGF1B is able to inhibit the activation of Smad2/3 [18]. There is a link between the disruption of the Smad2/3 pathway and the development of cancer [19]. Inactivation of Smad2/3 leads to the development of cisplatin resistance in osteosarcoma [20]. Cisplatin can perform its apoptosis-related activity in cancer cells via modifying ovarian carcinoma and increasing the formation of reactive oxygen species (ROS) [3]. Oncogenic cells have a greater capacity to respond to the anticancer drug cisplatin when Smad2/3 is activated [21]. The activation of Smad2/3 results in an increase in the synthesis of apoptosis-related proteins and a reduction in the activity of antiapoptotic proteins. Smad2/3 phosphorylation could be decreased in A2780-Res cells by either inhibiting miR-182A-3p or overexpressing TGF1B, whereas increasing Smad2/3 phosphorylation could be achieved by either silencing circ TYMP1 or overexpressing TGF1B. In experiments conducted on animals, suppressing miR-182A-3p reduced the formation of tumors, whereas overexpressing TGF1B led to an increase in the growth of tumors via ovarian carcinoma changing Smad2/3 phosphorylation.

The article "Circ TYMP1 Inhibits Carcinogenesis and Cisplatin Resistance in Ovarian Cancer by Reducing Smad2/3 Phosphorylation via a MicroRNA-182A-3p/TGF1B Axis" was retracted in 2023. Reasons: signs of a paper mill; suspected computer-generated content; unreliable results or conclusions; concerns about the data.

## 5. Conclusion

In ovarian carcinoma, circ TYMP1 stimulates the synthesis of TGF1B by sequestering miR-182A-3p and lowering Smad2/3 phosphorylation; this, in turn, enhances both carcinogenesis and cisplatin resistance. This work has the potential to contribute to the management of ovarian carcinoma, particularly ovarian carcinoma that is resistant to DDP. It is possible that circ TYMP1 and TGF1B are targets for ovarian carcinoma carcinogenesis and treatment resistance.

## Figures and Tables

**Figure 1:** Circ TYMP1 is highly expressed in ovarian carcinoma cells and tissues. RT-qPCR of ovarian carcinoma cell lines and IOSE80; (c) RT-qPCR of A2780 and drug-resistant A2780-Res cells. Three experiments exhibited standard deviation means. ^*∗*^*p*=0.05 when compared to adjacent/IOSE80/A2780. a, c, or a one-way ANOVA was utilized to analyze differences (b).

**Figure 2:** Silencing of circ_TYMP1 reduces drug resistance. In this study, we compared A2780 and cisplatin cells' survival rates, circ TYMP1 expression, and viability after different dosages of DDP, as evaluated by MTT. We also compared A2780-Res cells' capacity to form colonies, as determined by MTT. The mean SDs of three tests were provided. ^#^*p*=0.05 in comparison with sh-NC. We used one-way and two-way analysis of variance (ANOVA) to compare group B to groups D, E, and F (a, c).

The article "Circ TYMP1 Inhibits Carcinogenesis and Cisplatin Resistance in Ovarian Cancer by Reducing Smad2/3 Phosphorylation via a MicroRNA-182A-3p/TGF1B Axis" was retracted in 2023. Reasons: signs of a paper mill; suspected computer-generated content; unreliable results or conclusions; concerns about the data.

**Figure 3:** Circ_TYMP1 sponges miR-182A-3p. (a) The results of RT-qPCR, MTT, colony formation assay, and apoptosis assays were used to examine the expression of miR-182A-3p in A2780-Res cells transfected with a miR-182A-3p inhibitor. This study was performed using sh-circ TYMP1 + NC inhibitor and NC inhibitor (^*∗*^*p*=0.05). An ANOVA (a, d, e) was performed to compare the groups A, C, D, and E (b).

**Figure 4:** The roles of sh-circ_TYMP1 in A2780-Res cells to inhibit blovarian carcinomaks by miR-182A-3p. (a) The results of RT-qPCR, MTT, colony formation assay, and apoptosis assays were used to examine the expression of miR-182A-3p in A2780-Res cells transfected with a miR-182A-3p inhibitor. This study was performed using sh-circ TYMP1 + NC inhibitor and NC inhibitor (^*∗*^*p*=0.05). An ANOVA (a, d, e) was performed to compare the groups A, C, D, and E (b).

**Figure 5:** MiR-182A-3p directly binds to TGF1B. (a and b) and (c and d) show the relative levels of miR-182A-3p and TGF1B protein in ovarian carcinoma tumor and its surrounding tissues, respectively, as shown by luciferase assay (^*∗*^*p*=0.05 vs. NC mimic) and reverse transcription-quantitative polymerase chain reaction (RT-qPCR) and immunohistochemistry (IHC), respectively (^*∗*^*p*=0.05 vs. NC mimic). The mean standard deviation (SD) was calculated based on the average of three tests. C, D, G, H, I, and J were tested for differences using paired *t* tests, unpaired *t* tests, a one-way ANOVA, or a two-way ANOVA (b).

**Table 1:** Primer.

Symbol	Forward (5′-3′)	Reverse (5′-3′)
Circ_TYMP1	GCTGAGGTGACGGTCTCAAA	GCCTCCCAGTTTCATGGACA
TGF1B	ATCTGCGGCAAGGCGTTTTCCA	GAGCCCTCAGATTTGACCTGTC
GAPDH	GTCTCCTCTGACTTCAACAGCG	ACCACCCTGTTGCTGTAGCCAA

## Data Availability

Data are available on reasonable request from the corresponding author.
